The article "Sevoflurane Suppresses the Growth, Metastasis, and Invasion of Endometrial Carcinoma Cells via miR-195-5p/JAK2 Axis" was retracted in 2023. Reasons: signs of a paper mill; suspected computer-generated content; unreliable results or conclusions; concerns about the data.

# Sevoflurane Suppresses the Growth, Metastasis, and Invasion of Endometrial Carcinoma Cells via miR-195-5p/JAK2 Axis

**DOI:** 10.1155/2022/2398101

**Published:** 2022-02-22

**Authors:** Guowei Fu, Junlan Huang, Zhouquan Wu, Lin Zhao

**Affiliations:** ^1^The Affiliated Changzhou No.2 People's Hospital of Nanjing Medical University, Changzhou 213003, China; ^2^Changzhou Wujin Hospital of Traditional Chinese Medicine, Changzhou 213161, China

## Abstract

**Background:**

Highly invasive and destructive endometrioma is one of the most familiar primary malignant tumors among women. It has been studied that sevoflurane can influence the development of various malignancies. But whatever sevoflurane could influence endometrial tumors is unknown.

**Materials and Methods:**

Through CCK8 and transwell analysis, we investigated the influence of sevoflurane on the development of endometrial tumors in vitro. Then, we studied the function of miRNA-195-5p to promote sevoflurane to inhibit the development of endometrial tumors. Then, we predicted the target genes of miRNA-195-5p by online software and focused on JAK2. Through luciferase assay, we proved the direct binding and regulation of miRNA-195-5p to JAK2.

**Results:**

We showed that sevoflurane could inhibit the growth, metastasis, and invasion of endometrial tumors via miRNA-195-5p/JAK2 axis.

**Conclusions:**

Our research shows the function of sevoflurane in inhibiting the development of endometrial tumors via miRNA-195-5p/JAK2 axis. Our findings proved that sevoflurane is potentially beneficial for endometrial carcinoma patients with surgery and may be helpful for the choice of anesthetics in endometrial carcinoma operations.

## 1. Introduction

Endometrial carcinoma (EC) is one of the most familiar primary malignant tumors in North America [1]. In Asia, the prevalence of EC is increasing. EC prefers to occur in menopausal women and contributes to 4% of newly occurring cancer cases [2]. Surgery to remove cancer tissues with coming up chemotherapy and radiation is the most conventional treatment for EC [1]. But due to the resistance to chemotherapy and radiation, relapse of cancer results in a more than 95% 5-year mortality [3]. Recently, increasing studies revealed that the use of anesthetics could influence cancer cells and reduce the 5-year mortality of cancer patients [3, 4]. It has been shown that sevoflurane could inhibit the development of various cancers, including glioma, liver cancer, and other cancers [4–7]. But whatever sevoflurane could influence endometrial tumors has not been studied.

miRNA is a kind of small RNAs that widely participate in the cancer metabolism. It could influence the proliferation, apoptosis, differentiation, and other metabolism of the cancer cells [8]. Many miRNAs have been reported to inhibit the occurrence and development of tumors. It has been reported that miR-195-5p could suppress the development of EC [9]. Ding et al. found that inhibiting miR-1278 can reduce the growth, migration, and invasion of papillary thyroid cancer cells [10]. Researchers of different groups have observed that miR-195-5p in EC tissues was downregulated using bulk RNA sequencing [11–13]. Janus kinase 2 (JAK2) pathway is important in various biometabolisms [14]. Increasing evidence has been indicated that JAK2 may have a crucial role in tumor metastasis and invasion [15].

The article "Sevoflurane Suppresses the Growth, Metastasis, and Invasion of Endometrial Carcinoma Cells via miR-195-5p/JAK2 Axis" was retracted in 2023. Reasons: signs of a paper mill; suspected computer-generated content; unreliable results or conclusions; concerns about the data.

In this work, we found that sevoflurane inhibited EC cell proliferation, invasion, and migration via miR-195-5p/JAK2 axis. Our findings proved that sevoflurane is potentially beneficial for endometrial carcinoma patients with surgery and may be helpful for the choice of anesthetics in endometrial carcinoma operations.

## 2. Material and Methods

### 2.1. Cell Culture

Normal human endometrial epithelial cells, HEC1A, and Ishikawa were purchased from Lonza and cultured in DMEM medium (Lonza) containing 10% fetal bovine serum (Lonza).

### 2.2. Transfection

miR-195-5p inhibitor, NC inhibitor, miR-195-5p mimics, and miR-NC were obtained from Thermo Fisher Biotechnology. Transfection was performed using Lipo2000 (Thermo Fisher) according to the protocol of the manufacturer.

### 2.3. Treatment of Sevoflurane

Cells were cultured with sevoflurane at a concentration of 1%, 2%, or 4% for 4 h. Then, the cells were cultured at normal condition for 24 h and used for other experiments.

### 2.4. CCK-8 Proliferation

Cells were plated in 96-well plates with a concentration of 2000 cells per well. Then, the cells were performed with different treatments for 18 h at 37°C. Then, each well was added with 10 *μ*l CCK-8 reagent (Abcam) and cultured at 37°C for 1 h. A microplate reader (Thermo Fisher) was used for measurement, and the absorption values were used to calculate the cell viability.

### 2.5. Measurement of Cell Metastasis and Invasion

Transwell assay was used for determining the ability of cell metastasis and invasion.

For cell migration, invasion chambers which carry membrane with 8 *μ*m pores (Corning) were used for the assay. The upper chambers were seeded with cells in serum-free medium (BD Biosciences). The lower chambers were added with complete medium containing 10% FBS. After incubation at 37°C for 24 h, the cells in the lower chambers were fixed, stained with crystal violet solution, and counted using a microscope.

For cell invasion, the upper chambers were coated with Matrigel (BD Biosciences, Bedford, MA) before adding the cell suspensions.

The article "Sevoflurane Suppresses the Growth, Metastasis, and Invasion of Endometrial Carcinoma Cells via miR-195-5p/JAK2 Axis" was retracted in 2023. Reasons: signs of a paper mill; suspected computer-generated content; unreliable results or conclusions; concerns about the data.

### 2.6. RNA Isolation and qRT-PCR

We isolated the total RNA with Trizol (Invitrogen). cDNA library was constructed with an miRNA Reverse Transcription Kit (Qiagen). qPCR was performed on a CycleLighter (Roche), and the RNA levels of the target genes were normalized to those of GAPDH [16]. All the primers' sequences were listed as follows: GADPH Forward primer: AAGTATGACAACAGCCTCAAG; GADPH Reverse primer: TCCACGATACCAAAGTTGTC. JAK2 Forward primer: TCGGAAGGAAAAACAAGACAAG; JAK2 Reverse primer: TTTGTCGATGGTGGTGAAAAAC. miR-195-5p Forward primer: GCGCGTAGCTTATCAGACTGA; miR-195-5p Reverse primer: AGTGCAGGGTCCGAGGTATT.

### 2.7. Western Blot Analysis

Western blot was performed according to the previous work [17]. We got primary and secondary antibodies from Abcam. The bands were developed with an ECL kit (Thermo Fisher). The pictures were captured with ChemiDoc (Bio-Rad). The following primary antibodies were used: E-cadherin (ab1416), N-cadherin (ab18203), and GAPDH (ab8245).

### 2.8. Luciferase Reporter System

Dual-Glo Luciferase Assay System (Promega) was used. We introduced WT or mutant binding site sequences of JAK2 3′UTR (Figure 1(a)) into pmirGLO (Promega) was used for cotransfection of miR-195-5p mimics, and plasmids containing WT or mutant binding site were cotransfected into HEC1A or Ishikawa using Lipofectamine 2000 (Invitrogen). After culturing for 48 h, MicroLumatPlus LB96V luminometer (Berthold) was used for the analysis of the luciferase activity of the cells.

### 2.9. Statistical Analysis

Data are illustrated with a form of mean ± S.E.M. Analysis of significant differences between groups was calculated by SPSS using Tukey's test or two-tailed Student's *t*-tests. *P* < 0.05 was considered statistically significant.

## 3. Results

### 3.1. Sevoflurane Inhibits the Development of EC

We first proved that sevoflurane had no effect on normal human endometrial epithelial cells (Sup Figure 1). To detect if sevoflurane could affect the development of EC, HEC1A and Ishikawa cells were treated with different sevoflurane concentrations (1%, 2%, and 4%) for 4 h. CCK-8 analysis showed that the cell growth could be significantly reduced by sevoflurane in a dose-dependent manner (Figures 2(a) and 2(b)). Furthermore, transwell assay was performed to detect the influence of sevoflurane on EC cell metastasis and invasion. We found that the metastasis and invasion of EC cells could by dramatically suppressed by sevoflurane with a dose-dependent manner (Figures 2(c) and 2(d)). Combined the results above together, we investigated that the growth, metastasis, and invasion of EC cells could by vitally suppressed by sevoflurane in a dose-dependent manner. And according to the results, we chose 4% sevoflurane as the treatment concentration for the following study.

The article "Sevoflurane Suppresses the Growth, Metastasis, and Invasion of Endometrial Carcinoma Cells via miR-195-5p/JAK2 Axis" was retracted in 2023. Reasons: signs of a paper mill; suspected computer-generated content; unreliable results or conclusions; concerns about the data.

### 3.2. Sevoflurane Suppresses the Development of EC via miR-195-5p

It has been revealed that the development of EC cells could be suppressed by miR-195-5p [7]. Researchers of different groups have observed that miR-195-5p in EC tissues was downregulated using bulk RNA sequencing [8, 9, 11]. Therefore, we raised a hypothesis that sevoflurane may affect the growth, metastasis, and invasion of EC cells via miR-195-5p. Firstly, we confirmed that miR-195-5p expression in HEC1A and Ishikawa cells was reduced compared to normal human endometrial cells by qRT-PCR (Figure 3(a)). However, after treatment with 4% sevoflurane, miR-195-5p expression in HEC1A and Ishikawa cells was significantly increased compared to the control group (Figure 3(b)). Then, we knocked down miR-195-5p expression in HEC1A and Ishikawa cells and tested the relative features. We confirmed the knockdown efficiency of miR-195-5p inhibitors (Figure 3(c)). Furthermore, compared to the control group, significantly decreased ability of cell proliferation (Figure 3(d)), migration (Figure 3(e)), and invasiveness (Figure 3(f)) was observed after 4% sevoflurane treatment. Knocking down miR-95-5p expression could promote the growth, metastasis, and invasion of EC cells treated with sevoflurane when compared to cells treated with sevoflurane only (Figures 3(d)–3(f)). Thus, the inhibition function of sevoflurane on EC cell growth, metastasis, and invasion could be diminished by the knockdown of miR-195-5p. Those results above demonstrated that sevoflurane may function as an EC suppressor through the upregulation of miR-195-5p.

### 3.3. Direct Binding of mir-195-5p and JAK2

In order to explore whether JAK2 plays a key role in EC cells, we obtained the potential miRNA (miR-195-5p) that interacting with JAK2 3′UTR through the online software starbase, and we mutate the binding site of JAK2 3′UTR to miR-195-5p (Figure 1(a)). Compared with miR-NC transfection, the luciferase activity of JAK2-3′UTR-WT in EC cells could be suppressed by miR-195-5p overexpression (Figures 1(b) and 1(c)). However, miR-195-5p could not suppress the luciferase activity of JAK2-3′UTR-WUT compared with miR-NC (Figures 1(b) and 1(c)). Those above proved that miR-195-5p could directly regulate JAK2 mRNA through binding to JAK2 3′UTR. Furthermore, we confirmed that miR-195-5p overexpression could downregulate JAK2 expression in both mRNA and protein level compared to miR-NC (Figures 1(d) and 1(e)). Similarly, the expression of JAK2 in EC cells was significantly reduced in mRNA and protein levels with the treatment of sevoflurane (Figures 1(f) and 1(g)). These data indicated that miR-195-5p could reduce JAK2 expression by directly binding to the 3′UTR of JAK2 mRNA. Moreover, sevoflurane could suppress JAK2 expression through upregulating the expression of miR-195-5p.

The article "Sevoflurane Suppresses the Growth, Metastasis, and Invasion of Endometrial Carcinoma Cells via miR-195-5p/JAK2 Axis" was retracted in 2023. Reasons: signs of a paper mill; suspected computer-generated content; unreliable results or conclusions; concerns about the data.

### 3.4. Overexpression of JAK2 Rescue the Effect of Sevoflurane in EC Cells

Then, we investigated the effect of JAK2 on the suppression ability of sevoflurane on EC development. We overexpressed JAK2 in EC cells and confirmed JAK2 expression using Western blot (Figure 4(a)). However, the suppression function of sevoflurane on the growth, metastasis, and invasion of EC cells was vitally diminished by the overexpression of JAK2 (Figures 4(b)–4(d)). These findings profoundly indicated that overexpression JAK2 diminishes the effect of sevoflurane in EC cells.

## 4. Discussion

Of the female reproductive system, EC is one of the most familiar primary malignancies. Surgical removal of the primary foci and postoperative radiotherapy and chemotherapy are the most effective methods for treating endometrial cancer. However, due to the resistance to chemotherapy and radiation, relapse of cancer results in a more than 95% 5-year mortality [18]. Recently, increasing studies revealed that the use of anesthetics could influence cancer cells and reduce the 5-year mortality of cancer patients [18]. Several clinical studies have shown that anesthetics can influence the relapse of cancers after surgery; however, the mechanism behind the phenomenon is still unknown. Therefore, our research is aimed at exploring the influence of sevoflurane on EC, including the cell growth, migration, and invasion of EC cells.

Sevoflurane is a common anesthetic drug used in the treatment of tumors and has been shown to have antitumor effects. Sevoflurane is a kind of colorless, transparent, aromatic, and nonirritating liquid and can relax the airway smooth muscle. The road stimulation of sevoflurane is small, and the intraoperative hemodynamics was stable using sevoflurane [18]. Clinically, sevoflurane is used to maintain anesthesia no more than 4% [19]. Therefore, the concentration we used in this study is usual and safe. Our data about sevoflurane's toxicity on normal human endometrial epithelial cells also proved this. Early studies have shown that sevoflurane inhibited breast cancer cell proliferation by upregulating miR-203 [13]. Another study proved that sevoflurane could reduce the invasion of colorectal carcinoma cells by suppressing the formation of MMP-9 in lymphocytes [20]. In addition, sevoflurane acts on colorectal cancer, glioma, liver cancer, and other cancer cells and can inhibit cancer cell metastasis and invasion [3, 5, 6]. The findings of these studies revealed that sevoflurane could dramatically downregulated the proliferation, invasion, and metastasis of cancer cells.

miRNA is a class of endogenous regulatory noncoding RNAs which could directly bind to and degrade the target mRNAs [8]. Several groups have shown that sevoflurane may influence the expression of a set of genes in the endometrium [21]. Since miRNA plays an important role in regulating gene expression, so sevoflurane may induce the changes in gene expression which are mediated by miRNA. In our research, we have proved that miR-195-5p expression in EC cells was significantly increased after the treatment of sevoflurane. Double luciferase reporter gene detection revealed that miR-195-5p overexpression can inhibit luciferase activity of JAK2-3′UTR-WT in the cells. When the predicted JAK2 binding site was mutated, the suppressive function of miR-195-5p will disappear, thus confirming that JAK2 is the target of miR-195-5p. Our study is consistent with previous works, which illustrated that miR-195-5p was deceased in other cancers. Li et al. demonstrated that the tumor tissues of esophageal cancer patients had vastly lower miR-195-5p expression than that normal tissues [17]. Jiang et al. reported that miR-195-5p expression in tumor tissues of esophageal cancer patients was significantly reduced compared with normal tissues, while CDC42 expression was decreased [22].

The article "Sevoflurane Suppresses the Growth, Metastasis, and Invasion of Endometrial Carcinoma Cells via miR-195-5p/JAK2 Axis" was retracted in 2023. Reasons: signs of a paper mill; suspected computer-generated content; unreliable results or conclusions; concerns about the data.

In order to explore the influence of miR-195-5p on the biological effects of endometrial cancer, we overexpressed miR-195-5p in endometrial cancer cells. We observed that transfection of miR-195 mimics significantly decreased JAK2 expression and further inhibited the development of endometrial cancer, indicating that miR-195-5p exerts a suppressive effect, which may reduce the malignant biological characteristics of endometrial cancer cells by targeting JAK2. Li et al. demonstrated that transfection of miR-195-5p mimics in esophageal cancer EC109 and EC9706 cells can significantly increase miR-195-5p, downregulate its target gene HMGA2, and inhibit the proliferation activity of esophageal cancer cells EC109 and EC9706 [17]. Fu et al. revealed that transfection of miR-195 mimics dramatically decreased the proliferation activity of esophageal cancer cells Eca109 and TE13 and inhibited their clonal formation and invasion ability [23]. Zhao et al. showed that miR-195-5p targeting SOX4 can inhibit the epithelial-mesenchymal transition (EMT) in esophageal cancer cells and further suppress their metastasis and invasion [24]. Our study revealed that miR-195-5p could directly bind to JAK2 3′UTR and suppress JAK2 expression, attenuating the malignant biological features in endometrial cancer.

The article "Sevoflurane Suppresses the Growth, Metastasis, and Invasion of Endometrial Carcinoma Cells via miR-195-5p/JAK2 Axis" was retracted in 2023. Reasons: signs of a paper mill; suspected computer-generated content; unreliable results or conclusions; concerns about the data.

JAK/STAT pathway is widely participated in biological metabolisms, such as cell reproduction, differentiation, transformation, and immune regulation. Furthermore, JAK/STAT pathway is also involved in various cellular biological functions during tumorigenesis, such as apoptosis, metastasis, and invasion [25, 26]. JAK inhibitors can selectively inhibit JAK kinase, suppress JAK/STAT pathway, and serve as cancer suppressors. Our findings indicated that sevoflurane could act as a JAK inhibitor and downregulate JAK2 expression in mRNA and protein levels by enhancing miR-195-5p levels. Furthermore, sevoflurane intervenes JAK2 signaling pathway through the miR-195-5p/JAK2 axis in endometrial tumor cells. Knocking down miR-195-5p could restore JAK2-mediated tumor suppression of sevoflurane.

Taken together, sevoflurane could upregulate miR-195-5p expression, thereby inhibiting the JAK2 signaling pathway. These findings make a contribute to deeply understand the pharmacological effects of absorption of anesthetics and provide experimental basis for cancer patients to choose more reasonable anesthetics.

## Figures and Tables

**Figure 1:** miR-195-5p directly binds to JAK2 3′UTR. (a) Prediction of the binding sites of miR-195-5p and JAK2. (b, c) Luciferase reporter gene experiments were conducted in HEC1A and Ishikawa cells to verify the targeting relationship. (d, e) Detecting the expression level of JAK2 mRNA and protein after overexpression of miR-195-5p in HEC1A and Ishikawa cells. (f, g) Analysis of the mRNA and protein expression levels of JAK2 in HEC1A and Ishikawa cells after sevoflurane treatment using qRT-PCR. ^∗^*P* < 0.05, ^∗∗^*P* < 0.01, *n* = 3.

**Figure 2:** Sevoflurane inhibits endometrial tumor cell growth, metastasis, and invasion. (a, b) The CCK-8 analysis method was used to evaluate the proliferative ability of sevoflurane on HEC1A and Ishikawa cells. (c, d) The transwell test evaluated the influence of sevoflurane to the metastasis and invasion of HEC1A and Ishikawa cells. ^∗^*P* < 0.05, ^∗∗^*P* < 0.01, *n* = 3.

**Figure 3:** Sevoflurane suppresses the growth, metastasis, and invasion of EC cells via miR-195-5p. (a) The qRT-PCR method evaluated miR-195-5p expression in normal endometrial cells and endometrial cancer cells. (b, c) miR-195-5p expression in HEC1A and Ishikawa cells after treatment with sevoflurane and knockdown of miR-195-5p. (d) Exploring the influence of miR-195-5p knockdown on the growth of HEC1A and Ishikawa cells treated with sevoflurane using CCK-8 assay. (e, f) Exploring the influence of miR-195-5p knockdown on the metastasis and invasion of HEC1A and Ishikawa cells treated with sevoflurane using transwell assay. ^∗^*P* < 0.05, ^∗∗^*P* < 0.01, *n* = 3.

The article "Sevoflurane Suppresses the Growth, Metastasis, and Invasion of Endometrial Carcinoma Cells via miR-195-5p/JAK2 Axis" was retracted in 2023. Reasons: signs of a paper mill; suspected computer-generated content; unreliable results or conclusions; concerns about the data.

**Figure 4:** Overexpression JAK2 rescue the effect of sevoflurane in EC cells. (a) The efficiency of JAK2 overexpression in HEC1A and Ishikawa cells was examined by WB method. (b) The CCK-8 method was used to detect the differences between HEC1A and Ishikawa in different groups (con group, SEV group, SEV + JAK2 group), so as to compare the differences in cell proliferation. (c, d) Transwell experiment evaluated the changes of cell metastasis and invasion ability in different groups of HEC1A and Ishikawa (con group, SEV group, SEV + JAK2 group).

## Data Availability

The datasets used and/or analyzed during the current study are available from the corresponding author on reasonable request.

## Supplementary Materials

Supplementary Materials Supplementary Figure 1: sevoflurane has no effect on the cell viability of normal human endometrial epithelial cells.

## References

[1] Arora S., Balasubramaniam S., Zhang W. (2020). FDA approval summary: pembrolizumab plus lenvatinib for endometrial carcinoma, a collaborative international review under project Orbis. *Clinical Cancer Research*.

[2] Herreros-Villanueva M., Chen C. C., Tsai E. M., Er T. K. (2019). Endometriosis-associated ovarian cancer: what have we learned so far?. *Clinica Chimica Acta*.

[3] Gao C., Shen J., Meng Z. X., He X. F. (2020). Sevoflurane inhibits glioma cells proliferation and metastasis through miRNA-124-3p/ROCK1 Axis. *Pathology Oncology Research*.

[4] Fan L., Wu Y., Wang J., He J., Han X. (2019). Sevoflurane inhibits the migration and invasion of colorectal cancer cells through regulating ERK/MMP-9 pathway by up-regulating miR-203. *European Journal of Pharmacology*.

[5] Wang L., Wang T., Gu J. Q., Su H. B. (2018). Volatile anesthetic sevoflurane suppresses lung cancer cells and miRNA interference in lung cancer cells. *Oncotargets and Therapy*.

[6] Sun S. Q., Ren L. J., Liu J., Wang P., Shan S. M. (2019). Sevoflurane inhibits migration and invasion of colorectal cancer cells by regulating microRNA-34a/ADAM10 axis. *Neoplasma*.

[7] Yi W., Li D., Guo Y., Zhang Y., Huang B., Li X. (2016). Sevoflurane inhibits the migration and invasion of glioma cells by upregulating microRNA-637. *International Journal of Molecular Medicine*.

[8] Ramassone A., Pagotto S., Veronese A., Visone R. (2018). Epigenetics and microRNAs in cancer. *International Journal of Molecular Sciences*.

[9] Dai L., Yue Q., Wang H., Wang X. U., Li Y., Chen R. (2019). MiR-195 inhibits migration, invasion and epithelial-mesenchymal transition (EMT) of endometrial carcinoma cells by targeting SOX4. *Journal of Biosciences*.

The article "Sevoflurane Suppresses the Growth, Metastasis, and Invasion of Endometrial Carcinoma Cells via miR-195-5p/JAK2 Axis" was retracted in 2023. Reasons: signs of a paper mill; suspected computer-generated content; unreliable results or conclusions; concerns about the data.

[10] Ding W., Shi Y., Zhang H. (2021). Circular RNA circNEURL4 inhibits cell proliferation and invasion of papillary thyroid carcinoma by sponging miR-1278 and regulating LATS1 expression. *American Journal of Translational Research*.

[11] Gao X., Lu M., Xu W., Liu C., Wu J. (2019). miR-195 inhibits esophageal cancer cell proliferation and promotes apoptosis by downregulating YAP1. *International Journal of Clinical and Experimental Pathology*.

[12] Song L. R., Li D., Weng J. C. (2020). MicroRNA-195 functions as a tumor suppressor by directly targeting fatty acid synthase in malignant meningioma. *World Neurosurgery*.

[13] Luo J., Pan J., Jin Y., Li M., Chen M. (2019). MiR-195-5p inhibits proliferation and induces apoptosis of non-small cell lung cancer cells by targeting CEP55. *Oncotargets and Therapy*.

[14] Liu Z., Gan L., Zhou Z., Jin W., Sun C. (2015). SOCS3 promotes inflammation and apoptosis via inhibiting JAK2/STAT3 signaling pathway in 3T3-L1 adipocyte. *Immunobiology*.

[15] Gao J., Tian J., Lv Y. (2009). Leptin induces functional activation of cyclooxygenase-2 through JAK2/STAT3, MAPK/ERK, and PI3K/AKT pathways in human endometrial cancer cells. *Cancer Science*.

[16] Livak K. J., Schmittgen T. D. (2001). Analysis of relative gene expression data using real-time quantitative PCR and the 2−*ΔΔ*CT method. *Methods*.

[17] Li Y., Wu D., Wang P., Li X., Shi G. (2017). miR-195 regulates proliferation and apoptosis through inhibiting the mTOR/p70s6k signaling pathway by targeting HMGA2 in esophageal carcinoma cells. *Disease Markers*.

[18] Sun Q., Xu R., Xu H., Wang G., Shen X., Jiang H. (2017). Extracranial metastases of high-grade glioma: the clinical characteristics and mechanism. *World Journal of Surgical Oncology*.

[19] Purdon P. L., Sampson A., Pavone K. J., Brown E. N. (2015). Clinical electroencephalography for anesthesiologists: part I: background and basic signatures. *Anesthesiology*.

[20] Silber J., Lim D. A., Petritsch C. (2008). miR-124 and miR-137 inhibit proliferation of glioblastoma multiforme cells and induce differentiation of brain tumor stem cells. *BMC Medicine*.

[21] Hayase T., Tachibana S., Yamakage M. (2016). Effect of sevoflurane anesthesia on the comprehensive mRNA expression profile of the mouse hippocampus. *Medical Gas Research*.

[22] Jiang Y., Berry D. C., Tang W., Graff J. M. (2014). Independent stem cell lineages regulate adipose organogenesis and adipose homeostasis. *Cell Reports*.

[23] Fu M. G., Li S., Yu T. T. (2013). Differential expression of miR-195 in esophageal squamous cell carcinoma and miR-195 expression inhibits tumor cell proliferation and invasion by targeting of Cdc42. *FEBS Letters*.

The article "Sevoflurane Suppresses the Growth, Metastasis, and Invasion of Endometrial Carcinoma Cells via miR-195-5p/JAK2 Axis" was retracted in 2023. Reasons: signs of a paper mill; suspected computer-generated content; unreliable results or conclusions; concerns about the data.

[24] Zhao J., Li X., Yang Y. (2016). Effect of YAP1 silencing on esophageal cancer. *Oncotargets and Therapy*.

[25] Liu I. M., Schilling S. H., Knouse K. A., Choy L., Derynck R., Wang X. F. (2009). TGFbeta-stimulated Smad1/5 phosphorylation requires the ALK5 L45 loop and mediates the pro-migratory TGFbeta switch. *The EMBO Journal*.

[26] Cancer genome atlas research, N (2014). Comprehensive molecular characterization of gastric adenocarcinoma. *Nature*.

